The article "Context Aware Convolutional Neural Network for Children Caries Diagnosis on Dental Panoramic Radiographs" was published in 2022. Journal: Comput Math Methods Med.

# Context Aware Convolutional Neural Network for Children Caries Diagnosis on Dental Panoramic Radiographs

**DOI:** 10.1155/2022/6029245

**Published:** 2022-09-21

**Authors:** Xiaojie Zhou, Guoxia Yu, Qiyue Yin, Yan Liu, Zhiling Zhang, Jie Sun

**Affiliations:** ^1^Department of Stomatology, Beijing Children's Hospital, Capital Medical University, National Center for Children's Health, China; ^2^Institute of Automation, Chinese Academy of Sciences, China

## Abstract

The objective of this study is to improve traditional convolutional neural networks for more accurate children dental caries diagnosis on panoramic radiographs. A context aware convolutional neural network (CNN) is proposed by considering information among adjacent teeth, based on the fact that caries of teeth often affects each other due to the same growing environment. Specifically, when performing caries diagnosis on a tooth, information from its adjacent teeth will be collected and adaptively fused for final classification. Children panoramic radiographs of 210 patients with one or more caries and 94 patients without caries are utilized, among which there are a total of 6028 teeth with 3039 to be caries. The proposed context aware CNN outperforms typical CNN baseline with the accuracy, precision, recall, *F*1 score, and area-under-the-curve (AUC) being 0.8272, 0.8538, 0.8770, 0.8652, and 0.9005, respectively, showing potential to improve typical CNN instead of just copying them in previous works. Specially, the proposed method performs better than two five-year attending doctors for the second primary molar caries diagnosis. Considering the results obtained, it is beneficial to promote CNN based deep learning methods for assisting dentists for caries diagnosis in hospitals.

## 1. Introduction

Dental caries or called tooth decay is a prevalent infectious chronic dental disease, which is caused by the interaction of bacteria and sugary foods on tooth enamel [1]. Usually, if a child suffers from dental caries in the primary dentition, the probability of infections in the permanent dentition increases [2]. Due to above immediate and potential long-time damage to oral health, dental caries should be given enough attention in children oral health [3]. Fortunately, dental caries is preventable and once detected can be cured and may be reversed in the early stages [4].

X-ray radiography is one of the most important approaches that help radiologists to diagnose caries, especially for teeth that are hard to be detected by visual inspection [5, 6]. Generally, there are several popular dental x-rays that can be utilized for children caries detection [7–9], e.g., bitewing, panoramic, and periapical. Recently, panoramic radiography is widely utilized for dental caries diagnosis because of several advantages [10, 11]. Apart from a low radiation dose and high patient comfort, panoramic radiography consists of the entire patient dentition, based on which, caries can be diagnosed for each tooth in a single image [12].

However, panoramic radiographs of children are usually with primary or mixed dentition along with surrounding bones and jaw structure, making automatic caries diagnosis a hard problem [13]. To perform caries diagnosis on a panoramic radiography, there are often two possible steps [14, 15]: (1) extract all teeth to make a tooth isolate from others and (2) diagnose whether a tooth has decay. To extract teeth in panoramic radiographs, several works have been proposed based on conventional edge detection methods [16], genetic algorithms [17], and the most popular CNN networks [18–20]. The performance of tooth extraction is very important for caries recognition, and usually, a nurse or a trained data annotation worker could accomplish such step, so we move our focus on step two, which requires experience from expert dentist.

To perform caries classification on each tooth image, early studies extract statistical characteristics from the caries and normal tooth images and make a decision by discovering differences between them or by training classifiers. For example, Saravanan et al. [21] found that pixel intensities of caries and normal tooth are concentrated in different ranges, and spectrum of a decayed tooth has high frequency components in the spectral components compared with that of normal tooth. Virupaiah and Sathyanarayana [22] utilized Gaussian low pass filter to preprocess dental images, based on which, statistical features are extracted and used by support vector machine classifier for caries classification. Recently, with the breakthrough of deep learning [23, 24], especially its outstanding performances of image analysis based on CNN technology [25, 26], several works have been proposed for panoramic radiography caries diagnosis based on CNN [12, 14, 27–29].

Overall, most of previous CNN based panoramic radiography caries detection methods just utilize popular CNN architectures and put their focus on testing CNN performance or achieving efficient parameters transfer. For example, Vinayahalingam et al. [27] verified MobileNet V2 network on classifying caries of third molar. Bui et al. [14] tested the performance of several typical CNN frameworks on panoramic radiography caries detection, including Alexnet, Googlenet, VGG16, VGG19, Resnet18, Resnet50, Resnet101, and Xception networks. Haghanifar et al. [12] utilized CapsNet for binary caries classification and used transfer learning for feature extraction. To the best our knowledge, none of previous works consider a tooth caries predication using general knowledge of the field, e.g., information from its adjacent teeth, which we claim to be important because caries of teeth often affects each other due to the same growing environment.

Therefore, this study is aimed at proposing a novel context aware CNN for more accurate caries diagnosis of primary dentition on dental panoramic radiographs, by considering general knowledge of caries, i.e., collecting and adaptively fusing information from adjacent teeth to help diagnosis. Specifically, the proposed context aware CNN adopts a pooling strategy to collect information from adjacent teeth and utilizes an attention mechanism for current and adjacent teeth information fusion. Compared with conventional CNN frameworks, our method can be a plug-in component to improve those frameworks, based on which, those CNN frameworks can be enhanced to gather enough useful information for caries diagnosis. In summary, our method provides a framework to improve caries classification performance, which will be shown in the Results Section.

## 2. Materials and Methods

### 2.1. Ethics Statement

This study was conducted with the approval of the Institutional Review Board (IRB) of Beijing Children's Hospital, Capital Medical University, National Center for Children's Health (IRB No.: [2022]-E-044-R). This study was a noninterventional study, and no-clinical trail was performed.

### 2.2. Materials

This study was performed on panoramic radiographs of patients in Beijing Children's Hospital, Capital Medical University, National Center for Children's Health from December 2015 to December 2021. Patients diagnosed with one or more caries (decided by the diagnostic report) via panoramic radiograph were selected as part of the database. Besides, dental age-matched patients without caries (decided by five-years attending doctors) were selected from the same hospital and time period to serve as reference data. In total, there are 210 panoramic radiographs with at least one tooth caries and 94 without caries. In the above 304 panoramic radiographs, there are 6028 teeth, among which there are 3039 and 2989 teeth with and without caries, respectively. Note that some teeth are missing, but we keep those panoramic radiographs and just ignore those teeth positions. All panoramic radiographs are JPEG format with size around 2441 × 1150 pixels.

### 2.3. Methods

#### 2.3.1. Data Preprocessing

A panoramic radiograph consists of all the teeth, which should be extracted because dental diagnosis is usually performed for each individual tooth. Teeth extraction is out of the scope of this study, which can be accomplished by dentist, nurse, or trained data annotation workers. Based on several mature annotation tools such as via (https://www.robots.ox.ac.uk/vgg/software/via/), extracting each tooth is easily performed as shown in Figure 1.

It should be noted that teeth are diverse in shape and size, so we do not use the same sized rectangular box for all the teeth, leading to various input sizes for CNN model (tooth image should be resized before fed into CNN). Specially, when a tooth is missing in a panoramic radiograph, we leave it out of our database. After the tooth extraction process, we obtain a database consisting of all the teeth, based on which, we split the database into training, validation, and test sets. More details are summarized in Table 1.

#### 2.3.2. A Typical CNN Baseline

Resnet [30] is one of the most successful CNN architectures for image analysis, based on which, various computer vision tasks have reached state-of-the-art performance. Overall, Resnet utilizes residual block to alleviate gradient vanishing/exploding when increasing the number of layers, i.e., depth of the CNN. Recently, Resnet has been applied for caries diagnosis, and relatively good performance has been obtained [14]. In our model, Resnet (Resnet18 with 18 trainable layers) is utilized as a baseline method and a modular to form context aware CNN, which will be elaborated in the next subsection.

#### 2.3.3. Context Aware CNN

The aim of our proposed method is to improve caries classification performance. Considering teeth in the same mouth share the same growing environment, it is natural that if one tooth has dental caries, the probability of being caries of its adjacent teeth will be greatly increased. Based on such intuitive assumption, an idea of promoting caries classification performance is to encode the above information when developing CNN models. Accordingly, we propose a context aware CNN, and the overall framework is shown in Figure 2.

In the proposed model, there are three key steps: (1) current tooth and its adjacent teeth are fed into the Resnet model for higher level representations extraction; (2) representations of the adjacent teeth are merged through pooling operation to obtain an adjacent representation; and (3) current and adjacent representations are adaptively fused through attention network for final representation learning, based on which a classifier layer is adopted for final caries predication. Noted that we leave out the classifier layer of Resnet for high level representations extraction, and pooling is selected as average pooling.

Mathematically, suppose the higher level representations of the current tooth and its *k*_th_ adjacent tooth (using the same Resnet for representation extraction) are *r*_*c*_ and *r*_*ak*_, *k* = 1, ⋯, *K*, respectively, then, the adjacent representation *r*_*a*_ by merging all the *K* neighbors is calculated as

(1) $$\begin{array}{c} r_{a}=\text{pooling}\left(r_{a1},\cdots ,r_{aK}\right). \end{array}$$

By bringing in an extra multilayer perceptron network, we feed the network with concatenation of current and adjacent representations and obtain a weight *α* for the current representation based on sigmod activation function:

(2) $$\begin{array}{c} \alpha =\text{sigmod}\left(W_{2}\times \text{sigmod}\left(W_{1}\times \left(\left[r_{c},r_{a}\right]\right)+b_{1}\right)+b_{2}\right), \end{array}$$

where *W*_1_, *W*_2_, *b*_1_, and *b*_2_ are parameters of the multilayer perceptron network. Then, the final representation *r*_*f*_ of the current tooth is calculated by:

(3) $$\begin{array}{c} r_{f}=\alpha \times r_{c}+\left(1-\alpha \right)\times r_{a}. \end{array}$$

*r*_*f*_ will be fed into a softmax activated classifier layer for caries predication.

### 2.4. Network Training

In our database, there are 6028 teeth, which is big enough to train the deep neural networks, so we use no pretraining and just train the typical CNN baseline and our context aware CNN end to end. Contrast enhancement, adjusting the intensity of each pixel based on its relative magnitude with respect to the bilateral filter, is set to be 1.5 times, which we found is useful for caries classification. As for the data augmentation, we found no improvements can be obtained, so no data augmentation is utilized.

### 2.5. Training Configuration

The server used is configured with Intel(R) Xeon(R) Gold 6240R CPU and NVIDIA RTX 2080 Ti GPU (12GB ram), and the system is CentOS Linux release 7.8.2003. As for the hyperparameters, the network parameters are iterated for up to 10000 epochs using the Adam optimizer. The mini-batch size and the learning rate are set as 32 and 10^−3^, respectively. We select the model with the best performance on the validation set and then deployed to obtain the diagnosis results on the test set. Finally, the number of selected neighbors is set to be 3, and we will test the influence of varying numbers of neighbors in the following experiments.

### 2.6. Diagnostic Performance Evaluation

Similar with previous works, five classical metrics are adopted for performance evaluation, i.e., accuracy, precision, recall, *F*1-score, and AUC. We use TP, FP, FN, and TN to represent classification true positive, false positive, false negative, and true negative, respectively; then, the metrics are calculated as

(4) $$\begin{array}{c} \text{Accuracy}=\frac{\text{TP}+\text{TN}}{\text{TP}+\text{TN}+\text{FP}+\text{FN}}, \end{array}$$

(5) $$\begin{array}{c} \text{Precision}=\frac{\text{TP}}{\text{TP}+\text{FP}}, \end{array}$$

(6) $$\begin{array}{c} \text{Recall}=\frac{\text{TP}}{\text{TP}+\text{FN}}, \end{array}$$

(7) $$\begin{array}{c} F1=\frac{2\times \text{Precision}\times \text{Recall}}{\text{Precision}+\text{Recall}}. \end{array}$$

As for the AUC, it is the area under the receiver operating characteristic (ROC) curve. Noted for all the metrics, higher values represent a better performance.

## 3. Results

### 3.1. Diagnosis Performance

Table 2 details the caries classification performance of the proposed context aware CNN model and the typical CNN baseline. Due to the consideration of context information, our method outperforms the typical CNN baseline for about 5 to 7 percentages in terms of accuracy, precision, recall, and *F*1.  Figure 3 displays the ROC curves of the two methods with the area under the curve values, which again validates the helpfulness of utilizing context information for caries diagnosis.

To further verify the advantage of our proposed method, we show the classification accuracy for each tooth, as shown in Figure 4. It can be seen that our method outperforms the typical CNN baseline for most tooth positions. Specially, improvements against typical CNN baseline for teeth 54, 51, 63, 64, 65, and 81 are larger than 10 percentages, and up to about 17 percentage for tooth 71.

### 3.2. Parameter Sensitivity

In the proposed context aware CNN model, there is an important hyperparameter that controls how much context information is adopted. In this subsection, we change the neighbors selected to test the influence of this hyperparameter to the final performance.  Table 3 displays the results with neighbors selected as 2, 3, and 5, respectively. Taking tooth position 51 as an example, when the number of neighbors is 2, teeth 52 and 61 are selected; when the number of neighbors is 3, teeth 52, 61, and 81 are considered; when the number of neighbors is 5, teeth 52, 61, 81, 82, and 71 are selected. According to the results and Table 2, we can draw the following conclusions: (1) by considering the context information, caries classification performance can be improved no matter what the numbers of neighbors are selected (see CNN results in Table 2), and (2) when the number of neighbors is 3, best performance can be obtained. This is because with less neighbors considered, not enough information is utilized, but with much more neighbors selected, such information may cause extra complications.

### 3.3. Comparative Evaluation of the Abilities with Human

The diagnosis performance of human evaluators (two five-years attending doctors) and the proposed context aware CNN is presented in Table 4. It can be seen that the average classification performance of human evaluators is higher than that of the proposed method and the currently mainstream CNN baseline (see CNN results in Table 2). However, the time used for a panoramic radiograph image diagnosis of the proposed method is much less than that of human evaluators.

Table 5 displays the diagnosis accuracy of each tooth position for the proposed method and the attending doctors. Even through the attending doctors perform better in most tooth positions, the model works much better on primary molars like tooth positions 55, 64, 65, 75, and 85. One possible reason is that mild caries on primary molars is hard to be detected by human due to the lower contrast.

## 4. Discussion

With the breakthrough of deep learning, especially its outstanding performances in computer vision tasks based on CNN architecture, various advanced CNN approaches are developed. Benefited from the interdisciplinary study, researchers are borrowing the powerful CNN technology for stomatology imaging analysis. Very recently, CNN has been utilized for panoramic radiography caries detection, which is one of the most common diseases in oral health.

Various CNN methods have been tested for panoramic radiography caries classification, and relatively good performances have been obtained [12, 14, 27–29]. For example, Bui et al. [14] tested several typical CNN methods including the most famous Alexnet, Googlenet, VGG16, VGG19, Resnet18, Resnet50, Resnet101, and Xception networks. In their experimental results, values of accuracy, sensitivity, and specificity are 91.70%, 90.43%, and 92.67%, respectively. Based on the results, CNNs are promising for dentists and capable of wide-scale implementation caries detection in hospitals.

In this study, we aim to promote conventional CNN based methods for more accurate children caries diagnosis, so as to help clinical applications. The motivation lies in the observation that current deep learning based caries diagnosis approaches just copy the CNN methods designed for natural image analysis. We argue that the modality gap between natural image and dental panoramic radiographs image may cause performance degeneration, and most importantly, by properly considering general knowledge of caries classification may largely promote the diagnosis performance.

We propose context aware CNN by considering its adjacent teeth information when deciding whether a tooth is a caries. Specifically, the information of adjacent teeth is extracted utilizing the same networks used for the current tooth information extraction, and a three-layer perception network is adopted calculating weights for their adaptive fusion. Accordingly, only a small number of network parameters are added compared with conventional CNN frameworks. Results in terms of accuracy, precision, recall, *F*1, and AUC exceed typical CNN baseline. More specifically, the improvements are up to 5 to 7 percentages. We also display the diagnosis accuracy for each teeth position. Apart from three positions (61, 82, and 83), the proposed context aware CNN obtains much better performance with six positions (54, 51, 63, 64, 65, and 71) having at least 10 percentage improvements. The results show potential to revise current CNN approaches instead of just copying typical CNN methods for direct dental panoramic radiographs analysis.

In this study, we further validate the effects of the numbers of neighbors selected to form the context information. As neighbors of a tooth, we choose the neighbors based on the tooth positions. Taking tooth position 51 as an example: 2 neighbors means its left and right sides (positions 52 and 61); 3 neighbors will add its facing tooth (positions 52, 61, and 81); 5 neighbors will consider another two diagonal teeth (positions 52, 61, 81, 82, and 71). The results show that the best performance corresponds to 3 neighbors. This is reasonable, because those 3 neighbors are most close to the current tooth, which will largely help its diagnosis based on common sense. More or fewer neighbors considered may bring in noise information or ignore useful information, respectively.

The diagnosis abilities of human (five-years attending doctors) and the proposed method are compared. Almost all the evaluation metrics of the proposed context aware CNN are lower than that of the professional attending doctors, but the diagnosis speed of a dental panoramic radiograph image is significantly faster. More specifically, it takes an average of 1.0619 s for our context aware CNN model, but attending doctors need an average of 64.5000 s for a diagnosis of a dental panoramic radiograph image, showing a significant difference. So, if a deep learning based model is utilized for assisting caries diagnosis, it would help shorten the diagnosis time of clinicians especially for those with little experience. In the comparison of classification accuracy for each tooth, the proposed method outperforms professional attending doctors in the second primary molar. This is inspiring because it may provide a very useful auxiliary diagnosis for clinicians, such as to verify or improve the diagnosis accuracy on caries of the second primary molar.

This study also has some limitations. First, the proposed context aware CNN model is based on the extraction of each tooth from the dental panoramic radiographs, so extra human annotation is necessary, which limits its usage in clinical applications when performing computer aided diagnosis. Second, caries has different stages [28], so instead of making a binary classification of whether a tooth is a caries, it is more helpful to assist dentist to make an accurate diagnosis of what degree of the caries is. A follow-up study by considering different stages of caries and an end-to-end extraction and classification framework is necessary and will be studied in the future work.

## 5. Conclusions

By introducing general knowledge in the field to advance typical CNN model, a context aware CNN has been developed, which shows 5 to 7 percentage improvements compared with typical CNN baseline in terms of classification accuracy, precision, recall, *F*1, and AUC. The proposed model shows potential to revise typical CNN approaches instead of just copying them for direct dental panoramic radiographs analysis as in previous works. Furthermore, the results of this study are expected to help clinicians make decisions for children caries diagnosis on panoramic radiographs, especially for the second primary molar caries diagnosis, which shows higher accuracy than that of two five-year attending doctors.

## Figures and Tables

**Figure 1:** Extraction of each tooth on a panoramic radiograph.

**Figure 2:** Overall framework of the proposed context aware CNN.

**Figure 3:** Receiver operating characteristic (ROC) curves of the proposed context aware CNN (CA-CNN) and the typical CNN baseline (CNN). Numbers in parentheses show the area under the curve (AUC) values.

**Figure 4:** Classification accuracy of each tooth for our context aware CNN (CA-CNN) and the typical CNN baseline (CNN). Numbers in the horizontal ordinate denote the tooth positions.

**Table 1:** Data characteristics in this study.

Characteristics	Values
Total, with, and without caries panoramic radiograph numbers	304, 210, 94
Total, caries, and normal teeth numbers	6028, 3039, 2989
Training, validation, and test panoramic radiograph numbers	244, 30, 30
Training of total, caries, and normal teeth numbers	4833, 2432, 2401
Validation of total, caries, and normal teeth numbers	599, 320, 279
Test of total, caries, and normal teeth numbers	596, 287, 309

**Table 2:** Performance comparison between the proposed context aware CNN (CA-CNN) and the typical CNN baseline (CNN).

Methods	Accuracy	Precision	Recall	*F*1
CNN	0.7768	0.8056	0.8049	0.8052
CA-CNN	0.8272	0.8538	0.8770	0.8652

**Table 3:** Influence of the numbers of neighbors selected in the proposed context aware CNN (CA-CNN). CA-CNN-X means X neighbors being selected.

Metrics	Accuracy	Precision	Recall	*F*1	AUC
CA-CNN-2	0.8020	0.8051	0.8155	0.8103	0.8537
CA-CNN-3	0.8272	0.8538	0.8770	0.8652	0.9005
CA-CNN-5	0.8104	0.8452	0.8738	0.8593	0.8725

**Table 4:** Comparison of the classification performance and average testing time of a dental panoramic radiograph image between the proposed context aware CNN (CA-CNN) and two five-year attending doctors (AD, average performance is reported).

Metrics	Accuracy	Precision	Recall	*F*1	Time (s)
CA-CNN	0.8272	0.8538	0.8770	0.8652	1.0619
AD	0.8842	0.8509	0.9417	0.8940	64.5000

**Table 5:** Classification accuracy of each tooth for the proposed context aware CNN (CA-CNN) and two five-year attending doctors (AD, average performance is reported).

Position	55	54	53	52	51
CA-CNN	0.8333	0.8667	0.7000	0.7333	0.8667
AD	0.7667	0.9000	0.9333	0.9333	0.9333
Position	61	62	63	64	65
CA-CNN	0.7333	0.8000	0.8667	0.9667	0.9333
AD	0.8333	0.9333	0.8667	0.8667	0.8333
Position	75	74	73	72	71
CA-CNN	0.8621	0.9000	0.7667	0.8667	0.8276
AD	0.8276	0.9000	0.8333	1.0000	0.9310
Position	81	82	83	84	85
CA-CNN	0.8000	0.7667	0.7667	0.8621	0.8276
AD	0.9333	0.9000	0.9000	0.9310	0.7241

## Data Availability

Data used in this study were obtained from Department of Stomatology, Beijing Children's Hospital, Capital Medical University, National Center for Children's Health and are available with the permission of the Institutional Review Board (IRB) of Beijing Children's Hospital, Capital Medical University, National Center for Children's Health.
